The article "An Improved BERT and Syntactic Dependency Representation Model for Sentiment Analysis" was published in 2022. Journal: Comput Intell Neurosci.

# An Improved BERT and Syntactic Dependency Representation Model for Sentiment Analysis

**DOI:** 10.1155/2022/5754151

**Published:** 2022-05-05

**Authors:** Wenfeng Liu, Jing Yi, Zhanliang Hu, Yaling Gao

**Affiliations:** ^1^School of Computer, Heze University, Heze 274015, China; ^2^School of Computer Science and Technology, Shandong Jianzhu University, Jinan 250101, China

## Abstract

Text representation of social media is an important task for users' sentiment analysis. Utilizing the better representation, we can accurately acquire the real semantic information expressed by online users. However, existing works cannot achieve the best results. In this paper, we construct and implement a sentiment analysis model based on the improved BERT and syntactic dependency. Firstly, by studying the word embeddings of BERT, we have ameliorated the embeddings representation. Attention mechanism is added to the word embeddings, sentence embeddings, and position embeddings. Secondly, we have exploited the dependency syntax analysis of the text, and the dependency relationship of different syntactic components will be obtained. For different syntactic components, the hierarchical attention mechanism is used to construct the phrase embeddings or block embeddings. Finally, we splice the syntactic blocks for sentiment analysis. Extensive experiments show that the proposed model has a stronger ability than the baselines on two standard data sets.

## 1. Introduction

In recent years, with the popularization of social media such as WeChat, Face Book, Twitter, and Fetion, these media are changing people's lifestyles and habits. How to represent the text and understand their semantic information accurately is an important task. However, existing works cannot achieve the best results. In general, the composition of a text can be subdivided into paragraph-level, sentence-level, and word-level. The words are basic components, and the representation of text can be divided into a series of word combinations. Therefore, researching on the word-level representation is extremely important compared with the other two.

With the innovation of hardware technology, we can do a large number of calculations or parameter learning. However, how to integrate more semantic information on text representation is an important and difficult task for natural language processing. Harris has put forward an important idea on text representation as early as the 1950s, which is the famous distributed hypothesis: words with similar contexts have similar semantics. Firth elaborated Harris' thoughts a few years later. A more direct expression is that the semantic information about a word is mainly determined by its context. In the last ten years, the computing capability has been greatly improved, especially the wide application of GPUs and TPUs, which have made the analysis, calculation, and processing of big data easier.

The article "An Improved BERT and Syntactic Dependency Representation Model for Sentiment Analysis" was published in 2022. Journal: Comput Intell Neurosci.

The contributions of our paper are as follows:

1. We have improved BERT (iBERT) to obtain a better representation. Respectively, the Token Embeddings (TEs), Segment Embeddings (SEs), and Position Embeddings (PEs) have different attention weights.
2. We have constructed the syntax tree based on syntactic dependency of block embeddings.
3. Combining with the attention mechanism, we have constructed the embeddings representation of the text.

## 2. Related Works

The expression of any language can be divided into several levels, such as paragraph-level, sentence-level, and word-level. The basic unit of meaningful representation is word-level. There are two methods for the vectorized representation about words, one is the One-Hot model and the other is the Distributed Representation model.

The idea of One-Hot representation is very simple. The dimension of word embeddings is measured by the number of words appeared; that is, the dimension of each word is equal to the total number of words. Only the position where the word has appeared is represented by 1, and the remaining positions are represented by 0. For instance, the word embeddings of “computer” and “PC” are [0, 0, 1, 0, 0, 0, 0] and [0, 0, 0, 0, 0, 1, 0], respectively. As we all know, the two words have the same meaning. Nonetheless, the similarity between them is zero. Therefore, One-Hot representation cannot express the similarity of words. If the amount of data is increased, it is prone to dimension disasters. Therefore, many applications have adopted the Distributed Representation model.

### 2.1. Distributed Representation

To acquire the semantic information about words and alleviate a series of problems in depth, there are two classic models, Word2Vec and BERT. In 2003, Bengio et al. [1] proposed the NNLM model, which obtained the word embeddings when training and constructing a language model. On this basis, Mikolov et al. [2] proposed the Word2Vec which contained two models (Continuous Bag-of-Words and Skip-gram) in 2013. The CBOW model used the context to predict the current word, while the SkipGram model used the current word to predict the context.

In 2018, Devlin et al. [3] proposed the BERT model (Bidirectional Encoder Representations from Transformers), which is another substantial achievement after Word2Vec. And it has achieved the optimal results on 11 tasks in natural language processing. This achievement also proved the importance of the two-way and pretraining model for text representation. Many related models have appeared one after another, such as SpanBert [4], RoBERTa, and XLNet [5]. To further improve the text language processing effect, a convolutional neural network model, Hybrid convolutional neural network (CNN), and Long Short-Term Memory (LSTM) based on the fusion of text features and language knowledge were proposed [6]. Chen et al. [7] proposed a new representation learning method combined with variational autoencoder (VAE) and density-based spatial clustering of applications with noise (DBSCAN).

The article "An Improved BERT and Syntactic Dependency Representation Model for Sentiment Analysis" was published in 2022. Journal: Comput Intell Neurosci.

### 2.2. Coarse-Grained Semantic Representation

Combining textual semantics, we can construct larger granularity of text representation, such as grammatical blocks, sentence-level, and document-level. The Paragraph Embeddings [8] and the Skip-Thoughts were the influential models. Paragraph Embeddings consisted of two submodels. One was to evaluate the central word-by topic embeddings and context information. The other used paragraph or sentence level evaluated the probability of words. However, Skip-Thoughts had an integrated encoder and decoder which modeled the context-related topics of physically adjacent sentences.

Furthermore, to achieve accurate semantic information in multiple documents, Lin et al. [9] proposed a semantic search model for knowledge documents. Yan and Gao [10] studied the coupling of internal topics and topological structure, and they modeled large-grained semantics. Wu et al. [11] proposed a multigranularity and cross-text semantic matching method by a deep neural network, which had obtained better results in the text matching field.

In recent years, due to the wide application of deep learning in text processing, the combination of multiple models (such as RNN, CNN, LSTM, GRU, Transformer, and BERT) is very widely used. Sun et al. [12] proposed a secure indoor crowdsourced localization system, BERT-ADLOC, which was based on BLE fingerprints. The system consisted of two main parts: adversarial sample discriminator BERT-AD and indoor localization model BERT-LOC. Jiang and He [13] had presented an attention mechanism that differentiated the focus on the output of ResNet and the long short-term memory for the features of the sequences. Alahmadi et al. [14] proposed a smartphone-based periocular recognition which used a deep convolutional neural network and collaborative representation. Cross-modal convolution could enable the use of efficient CNN-style layers for multimodal sequential models.

In addition, other models which have obtained excellent performance in image fields have been gradually migrated and applied to some subtasks of text processing. The convolutional models, which have combined words and phrases, have achieved better results in classification and sentiment analysis [15].

The article "An Improved BERT and Syntactic Dependency Representation Model for Sentiment Analysis" was published in 2022. Journal: Comput Intell Neurosci.

## 3. The Text Representation Model of Online Social Media

Any language has its corresponding language features and grammatical rules which are the key requirements for the meaningful expression. Therefore, making use of the word embeddings and grammatical structure, we can construct a better semantic representation of the text. Firstly, given a text in social media, it is necessary to preprocess the text (such as word segmentation and part-of-speech). Secondly, we have proposed the improved BERT model to obtain better word embeddings and utilized the direct dependencies of words to build a dependency tree. Finally, the improved BERT model (iBERT) and dependency trees are used to construct the semantic representation of the text. The framework is shown in Figure 1.

### 3.1. Word Embeddings Based on the iBERT

BERT obtains the input embeddings by summing multiple embeddings. These embeddings include the Token Embeddings (TEs), Segment Embeddings (SEs), and Position Embeddings (PEs). We have improved the BERT. The final inputs are represented by attention summation of the three embeddings, as shown in the following equation:

(1) $$\begin{array}{c} {\text{Input}}_{\text{EmbeddingsBERT}}=\alpha *E_{\text{TE}}+\beta *E_{\text{SE}}+\gamma *E_{\text{PE}}, \end{array}$$

where *α*, *β*, and *γ* are the attention weights of TE, SE, and PE.

As shown in Figure 2, *E*_TE_ ∈ *ℝ*^*N∗d*_model_^, *E*_PE_ ∈ *ℝ*^*N∗d*_model_^, *N* is the length of the input sequence, and *d*_model_ is the dimension of the word embeddings.

Position Embeddings *E*_0_, *E*_1_, *E*_2_, *E*_3_,…, *E*_*n*_ are obtained by equations (2) and (3). To facilitate comparison with the standard BERT, our paper adopts the same formulas as the official.

(2) $$\begin{array}{c} E_{\text{PE}\left(\text{pos},2i\right)}=\sin\left(\frac{\text{pos}}{\left(10000^{2i/d_{\text{model}}}\right)}\right), \end{array}$$

(3) $$\begin{array}{c} E_{\text{PE}\left(\text{pos},2i\right)}=\cos\left(\frac{\text{pos}}{\left(10000^{2i/d_{\text{model}}}\right)}\right), \end{array}$$

where pos denotes the position number of the word in the input sequence. The word in the even position is calculated by equation (2) (in the odds by equation (3)).

The overall framework of the BERT model utilizes the officially released structure. Transformer that belongs to the encoder-decoder architecture uses a two-way and self-attention mechanism. The main operations of the encoder in Transformer module are the following equations:

(4) $$\begin{array}{c} e_{\text{mid}}=\text{ayer Norm}\left(e_{in}\right)+\text{Multi Head Attention}\left(e_{\text{in}}\right), \end{array}$$

(5) $$\begin{array}{c} e_{\text{out}}=\text{Layer Norm}\left(e_{\text{mid}}+\text{FFN}\left(e_{\text{mid}}\right)\right), \end{array}$$

where *e*_in_ ∈ *ℝ*^*N∗d*^ denotes the input of the encoder and *e*_out_ ∈ *ℝ*^*N∗d*^ denotes the output of the encoder. Multi Head Attention(·) represents a multiheaded attention mechanism. FFN(·) is a feedforward neural network. Layer Norm(·) represents layer normalization.

The article "An Improved BERT and Syntactic Dependency Representation Model for Sentiment Analysis" was published in 2022. Journal: Comput Intell Neurosci.

In the Transformer module of iBERT, the main operations of the decoder are as follows:

(6) $$\begin{array}{c} d_{\text{mid}1}=\text{LayerNorm}\left(d_{\text{in}}+\text{MaskedMultiHeadAttention}\left(d_{\text{in}}\right)\right),\\ d_{\text{mid}2}=\text{LayerNorm}\left(d_{\text{mid}1}+\text{MaskedM}\_H\_\text{Attention}\left(d_{\text{mid}1},e_{\text{out}}\right)\right),\\ d_{\text{out}}=\text{LayerNorm}\left(d_{\text{mid}2}+\text{FFN}\left(d_{\text{mid}2}\right)\right), \end{array}$$

where *d*_in_ ∈ *ℝ*^*M∗d*^ denotes the input of the decoder. *d*_out_ ∈ *ℝ*^*M∗d*^ denotes the output of the decoder. Multi Head Attention(·), Layer Norm(·), and FFN(·) represent the same functions as those of the encoder. Masked Multi Head Attention(·) is a masked and multihead attention mechanism.

### 3.2. Syntax Tree Construction Based on Syntactic Dependency

The syntactic tree of a sentence is an interdependence graph of its words which determine their importance by the distance from the central word. Andor et al. [16] proposed a transformation-based dependency syntax analysis method. And they developed the SyntaxNet (http://github.com/tensorflow/models/tree/master/syntaxnet) system, which was the most popular construction method of the syntax tree. Through researching this system and making corresponding improvements, we have adopted a generation scheme for the syntax tree based on the arc transformation. This method uses a stack (STACK), buffer (BUFFER), and set (ARC_SET) [17]. *s*_1_*s*_2_…*s*_*j*_*…s*_*n*_ is a given text; *s*_*j*_ is the *j*th word. The execution is that the STACK only has the root node at the beginning. The ARC_SET is an empty set, while the BUFFER saves the word sequence of input. There are three operations, LEFT_ARC, RIGHT_ARC, and SHIFT (see Algorithm 1). The LEFT_ARC operation is that the current word in the buffer will be added a left arc to the word on top of stack, the RIGHT_ARC operation will add a right arc as LEFT_ARC does, and the SHIFT operation will transfer the current word into stack. Until all words in the buffer are all processed, the state of STACK is consistent with the initial, and the construction of the syntax tree has been completed.  Figure 3 is the dependency tree constructed by this method of the sentence “a woman washed the dishes.”

The article "An Improved BERT and Syntactic Dependency Representation Model for Sentiment Analysis" was published in 2022. Journal: Comput Intell Neurosci.

### 3.3. Text Representation Based on iBERT and Syntactic Dependence

The dependency tree is constructed by Algorithm 1. According to the different attention weights in different syntactic positions, we combine and splice them into the corresponding text semantic representation. For a sentence *S* = [*s*_1_, *s*_2_,…, *s*_*i*_,…, *s*_*n*_], *s*_*i*_ is the *i*-th word of sentence *S*. Embeddings (*s*_*i*_) represents the word embeddings obtained by iBERT, and Attentions (*s*_*i*_) is the weight of *s*_*i*_ obtained by grammatical analysis. It satisfies the normalization, as shown in the following equation:

(7) $$\begin{array}{c} \sum_{i=1}^{n}\text{Attentions}\left(s_{i}\right)=1. \end{array}$$

Combining the attention mechanism and word embeddings, we construct sentence embeddings, as shown in equation (8). Attentioned_Embeddings_*s*_*i*__ is abbreviated as *A*_*E*_*s*_*i*__.

(8) $$\begin{array}{c} A\_E_{s_{i}}=\text{Embeddings}\left(s_{i}\right)*\text{Attentions}\left(s_{i}\right). \end{array}$$

According to the constructed syntactic tree, which contains the dependency relationship between words, we can construct the phrase embeddings of the syntax blocks (equations (9) and (10)). The phrase embeddings are attention_weighted of their words, as shown in Figure 4. Where Represent_sentence_ denotes the semantic embeddings and phrase_vector_*i*__ represents the syntactic elements in the sentence which are mainly involving the subject, predicate, object, and other syntactic elements.

(9) $$\begin{array}{c} {\text{phrase}}_{\text{vector}\_m}=\frac{1}{k}*\sum_{j}A\_E_{j}. \end{array}$$

(10) $$\begin{array}{c} {\text{Represent}}_{\text{sentence}}=\left[{\text{phrase}}_{{\text{vector}}_{1}},\ldots ,{\text{phrase}}_{{\text{vector}}_{i}}\text{,}\ldots ,{\text{phrase}}_{{\text{vector}}_{p}}\right], \end{array}$$

### 3.4. The Sentiment Analysis Model Based on iBERT and Syntactic Dependency

To verify the effectiveness of the proposed model, we construct a text sentiment model in this section, as shown in Figure 5.

We denote the text embeddings as Text*_*1, Text_2,…, Text*_n*. The stage from the vectorized representation to the sentiment categories is a fully connected network. Parameter weight *W* is obtained after training, and this matrix is locked (or fixed) during the test. Sentiment categories *C*={*c*_1_, *c*_2_,…, *c*_*k*_}. *k* is the total number of categories in the sentiment classification, and the probability *P*_*c*_ that belongs to a certain category is obtained by the following formula:

(11) $$\begin{array}{c} P_{c}=W\cdot \text{TE}\\ =\left\{P_{c_{1}},P_{c_{2}},\ldots ,P_{c_{k}}\right\}. \end{array}$$

We use the softmax function to normalize and obtain the category with the highest probability, as shown in the following equation:

(12) $$\begin{array}{c} P_{c_{\max}}=\text{softmax}\left\{P_{c_{1}},P_{c_{2}},\ldots ,P_{c_{k}}\right\}. \end{array}$$

The cross-entropy Loss_*i*_ is used to train the model, and the formula is shown in the following equation:

(13) $$\begin{array}{c} {\text{Loss}}_{i}=-\frac{1}{k}\sum_{m}y_{\text{im}}\log\left(P_{c_{\text{im}}}\right), \end{array}$$

where *y*_*im*_ represents the probability that the *i*-th sample belongs to the *m*-th class (*m* ∈ *C*). If it belongs to the *m*-class, *y*_*im*_ is 1; otherwise, it is zero. *P*_*c*_*im*__ represents the prediction probability of the *i*-th sample belonging to the *m*-th category. To ensure obtaining a more robust model, we have utilized a dropout strategy. The dropout is used in a fully connected network with the vectorized representation TE to sentiment category *C*, and the value of dropout is set to 0.5.

The article "An Improved BERT and Syntactic Dependency Representation Model for Sentiment Analysis" was published in 2022. Journal: Comput Intell Neurosci.

## 4. Experiments and Results

### 4.1. Data Set and Evaluations

#### 4.1.1. Data Set

The first data set is task 4 in SemEval 2014, which contains two subdata sets, one is the Laptop and the other is the Restaurant. Their format is described by XML. In the Laptop, the number of sentences in training is 3045 and in the test is 800. In the Restaurant, the number of sentences in training is 3041, and the number of sentences in the test is 800.

Another data set is Subtask A [18] in SemEval 2017, which is mainly used for SDQC support and rumor classification. The classification of the training or testing is shown in Table 1.

*S*, *D*, *Q*, and *C,* respectively, represent the four categories, which are the support category (Support), the objection category (Deny), the doubt category (Query), and the irrelevant comment category (Comment). Category *S* denotes supporting related content. Category *D* represents the opposing related content. Category *Q* owns questions about related content, and category *C* expresses comments that have nothing to do with related content or themes.

#### 4.1.2. Evaluation

We have used the accuracy (AC) for evaluation of the experiments as shown in the following equation:

(14) $$\begin{array}{c} \text{AC}=\frac{\text{TP}+\text{TN}}{\text{TP}+\text{TN}+\text{FP}+\text{FN}}. \end{array}$$

TP (True Positive) indicates that the predicted (positive) is consistent with the actual (positive). FP (False Positive) denotes that the predicted (positive) is inconsistent with the actual (negative). TN (True Negative) represents that the predicted (negative) is consistent with the actual (negative). FN (False Negative) indicates that the predicted (negative) is inconsistent with the actual (positive).

The article "An Improved BERT and Syntactic Dependency Representation Model for Sentiment Analysis" was published in 2022. Journal: Comput Intell Neurosci.

### 4.2. Parameter Settings

In the learning stage of word embeddings, the number of layers used is 12 (num_hidden_layers = 12). The number of neurons in the hidden layer of the neural network is 768 (hidden_size = 768), and the length of the input text is uniformly set to 512 characters (num_hidden_layers = 512), the dropout is set to 0.1 (attention_probs_dropout_prob = 0.1), the activation function that used is gelu function (hidden_act = “gelu”), and the number of parameters is about 110 M.

During the construction of the syntactic tree, we use the default parameters in the SyntaxNet system, the small batch size of the syntax analyzer is 32 (parser_batch_size = 32), the learning rate is 0.08 (learning_rate = 0.08), and the momentum is 0.85 (momentum = 0.85)).

### 4.3. Baselines

The comparison models are as follows:

1. TLSTM [19] divides words into two subsequences, one subsequence is from left to right and the other is from right to left, so two different embeddings will be obtained. The two embeddings coalesce into the final embeddings.
2. Att-LSTM [20] has utilized the attention mechanism in which the words have different attention weights. The text representation is constructed by the weighted words.
3. CABSA [21] combines the cyclic neural network, RNN, attention mechanism, and the memory network to acquire the representation through different directions in the sentence.
4. AGCN [22] uses two gated-based convolutional neural networks. They can obtain different representations, and the gated mechanism can learn the relational information of words.
5. BERT [3] utilizes the transformer as a submodule and obtains word embeddings by a two-way mechanism.
6. GCNDA [23] obtains the weight of words by combining the graphed attention mechanism, and it has two attentions, global and local.

Since there are fewer available comparison models in Subtask A, this paper uses eight models in the system which are released for comparison experiments.

### 4.4. Experiment Results

#### 4.4.1. Parameters *α*, *β*, and *γ*

*α*, *β*, and *γ*, which, respectively, denote the parameters of word embeddings, sentence embeddings, and position embeddings, take the same value in the iBERT model. For better verifying the effects, we have fixed one parameter and adjust the other two. Task_1 in BERT is used for measurement between the new embeddings and the standard word embeddings. During the experiments, the parameters are normalized by *α* + *β* + *γ* = 1.

For example, *α* is {0, 0.2, 0.4, 0.6, 0.8, 1}. *β* is fixed to 1, and *γ* is {1, 0.8, 0.6, 0.4, 0.2, 0}, respectively. After normalization, the values of parameter *α* are {0, 0.1, 0.2, 0.3, 0.4, 0.5}, *β* is 0.5, and *γ* is {0.5, 0.4, 0.3, 0.2, 0.1, 0}. The settings of the three parameters are shown in Table 2.

The article "An Improved BERT and Syntactic Dependency Representation Model for Sentiment Analysis" was published in 2022. Journal: Comput Intell Neurosci.

As shown in Figures 6(a)–6(c), the parameters alpha, beta, and gamma refer to *α*, *β*, and *γ*, respectively. After in-depth analysis of the composition of embeddings, the weight of the word is relatively high, followed by the sentence embeddings and the position embeddings. With fixed position embeddings, the final effect is gradually improved, and the main reason is that part of the word information is contained in the sentence embeddings. The composition of the sentence embeddings can be regarded as embeddings with larger granularity. And all words in the same sentence are used with the same sentence embeddings. To a certain extent, it weakens the representation of word embeddings in the same sentence. However, from another perspective, the word embeddings added to the sentence have a degree of distinction between sentences. Therefore, the sentence embeddings are meaningful in the sentence representation. Simultaneously, the calculation of the position embeddings is obtained by equations (2) and (3), which is the empirical formula of BERT team. The main reason is that the different position has different weights for the composed embeddings. After a number of experimental analyses, when *α*, *β*, and *γ* are, respectively, 0.65, 0.20, and 0.15, better word embeddings can be obtained.

#### 4.4.2. Experimental Results on SemEval 2014

From the results in Table 3 and Figure 7, we can get the following conclusions. The TLSTM model has the lowest accuracy among all baselines. The main reason is that this model only considers part of the content and ignores the representation of deep features. The Att-LSTM model can capture the deep features through the long short-term memory network. Simultaneously, it combines the attention mechanism to obtain the relationship of words in different locations. Hence, this model is more accurate than the TLSTM model. The CABSA model uses a memory network, and the effect of memory-based network is better than seq2seq-related models. The CABSA model can memorize the preceding or subsequent text feature through the memory network. So, this method has achieved a certain improvement to the previous two models.

Because the AGCN model has used two gated convolutional networks, the relationship of words can be obtained to a certain extent, but the syntactic structure cannot be captured commendably. Since BERT is an excellent and pretraining model in recent years, expression ability of word embeddings can be optimized, but the word embeddings constructed by the addition of embeddings can weaken the characteristic information such as syntactic structure. The GCNDA model is the best model among the baselines. The main reason is that this model has used a graphed convolution and combined with an attention mechanism, so that this model can obtain part of the structured information.

The article "An Improved BERT and Syntactic Dependency Representation Model for Sentiment Analysis" was published in 2022. Journal: Comput Intell Neurosci.

Our proposed model is BDPT, which combines the improved BERT and the syntactic structure. It has used the attention mechanism and combined syntactic blocks to construct a combinative text representation. Therefore, our method can obtain a deep-level representation of semantic information, and it has achieved higher precision in the classification task of sentiment analysis. Compared with the best model in baselines, our model has improved by 2.1% on the Restaurant and 1.9% on the Laptop.

Specifically, the time (seconds per ten sentences) consumed by BDPT is also the lowest (in Figure 8). Through in-depth analysis, the time complexity of TLSTM is *O*(*n∗m* + *n∗n* + *n*), *n* denotes Hidden_size, and *m* represents input_size. Att-LSTM adds a weight matrix, and the time complexity is *O*(*n∗m* + *n∗n* + *n* + *a∗*a), a denotes the attention weight matrix. AGCN is equivalent to having two gates, and it is close to double times of TLSTM. GCNDA adopts a four-layer network structure and involves the relationship matrix between words, so the time consumption is close to CABSA. Among all the comparison models, BERT has the lowest time complexity. The main reason is that its pretraining time is not taken into account.

#### 4.4.3. Results on SemEval 2017

Results on SemEval 2017 are shown in Table 4 and Figure 9. The DFKI_DKT model only uses sparse word embeddings as input, which has achieved the worst effect among all comparison models. The IITP model uses pairs of the original text and its response as the input. The IKM model uses the convolutional neural network to obtain the text representation, and it uses the softmax classifier to assign the probability that each category belongs to. IITP and NileTMRG are implemented by linear and polynomial kernel classifiers, respectively, while they are less effective. The MamaEdha model has mixed and used a variety of neural networks as classifiers. The ECNU system has solved the problem of information imbalance by decomposing it into a two-step classification task. DFKI-DKT, MamaEdha, ECNU, and UWaterloo use integrated classifiers, and the results of the classification are obtained through a voting mechanism. The three models, DFKI-DKT, ECNU, and MamaEdha, use the mixture of deep learning, machine learning, and manual rules to assign different labels with different weights.

The article "An Improved BERT and Syntactic Dependency Representation Model for Sentiment Analysis" was published in 2022. Journal: Comput Intell Neurosci.

All these compared models have used carefully designed feature engineering. IITP, NileTMRG, ECNU, and UWaterloo have utilized keywords and key sentences, as well as features in the Tweet (such as metadata, tags, and keywords for specific events). IKM and MamaEdha have used fewer features and exploited the word embeddings obtained from the CCN network.

The Turing model uses the LSTM network to implement sequence-to-sequence classification. This model comprehensively considers the word embeddings, punctuation embeddings, and the similarity between words, and it has incorporated more feature information. Consequently, it has obtained the best result in baselines. Compared with all the baselines, our proposed method has incorporated more in-depth features (such as improved BERT and syntactic dependency trees). And it has achieved the better result (1.5% higher than the best baseline). Further, our model has a better representation than all of them because syntactic structure plays a very important role in the text representation too. At the same time, our model takes the least amount of processing time.

## 5. Conclusions and Future Work

How to represent the text better is an important task in data mining and data analysis. This paper combines the existing research results and conducts a further study. In addition, we have proposed a novel model which has combined the improved BERT and grammatical dependency structure. Incorporating the deep semantic features into text representation, we can obtain a better sentiment analysis model. First of all, we have constructed a better text representation by studying the grammatical structure and iBERT. Then, we construct the syntactic dependency graph of words. Finally, extensive experiments have been performed on SemEval 2014 and SemEval 2017. Our model has achieved the state-of-art. Experiments show that syntactic structure plays an essential role in the text representation. The next step is to combine more deep-level features (such as the syntactic structure combined graph convolutional neural networks) for researching text and image sentiment analysis.

## Figures and Tables

**Figure 1:** The proposed model.

**Figure 2:** The improved word embeddings model.

**Figure 3:** An example of a syntactic tree.

**Figure 4:** The block embeddings of Syntactic tree.

**Figure 5:** The sentiment analysis model.

**Figure 6:** Experimentson *α*, *β*, and *γ*: (a) fix *α*; (b) fix *β*; (c) fix *γ*.

**Figure 7:** Model comparison diagram.

**Figure 8:** Elapsed time for different models.

**Figure 9:** Results on SemEval 2017 (Subtask A).

**Algorithm 1:** ARC_model ().

**Table 1:** The number of training and testing on SemEval 2017.

	*S*	*D*	*Q*	*C*

Training	910	344	358	2907
Testing	94	71	106	778

The article "An Improved BERT and Syntactic Dependency Representation Model for Sentiment Analysis" was published in 2022. Journal: Comput Intell Neurosci.

**Table 2:** Experiments of parameters *α*, *β*, and *γ*.

Group_1			Group_2			Group_3		
*α*	*β*	*γ*	*α*	*β*	*γ*	*α*	*β*	*γ*

0.5	0	0.5	0	0.5	0.5	0	0.5	0.5
0.5	0.1	0.4	0.1	0.5	0.4	0.1	0.4	0.5
0.5	0.2	0.3	0.2	0.5	0.3	0.2	0.3	0.5
0.5	0.3	0.2	0.3	0.5	0.2	0.3	0.2	0.5
0.5	0.4	0.1	0.4	0.5	0.1	0.4	0.1	0.5
0.5	0.5	0	0.5	0.5	0	0.5	0	0.5

**Table 3:** The accuracy on the Restaurant and Laptop.

Model	Restaurant	Laptop

TLSTM	0.752	0.668
Att-LSTM	0.761	0.672
CABSA	0.771	0.687
AGCN	0.772	0.688
BERT	0.782	0.694
GCNDA	0.789	0.702
**BDPT**	**0.810**	**0.721**

**Table 4:** Results on SemEval 2017 (Subtask A).

Models	AC

DFKI_DKT	0.635
IITP	0.641
IKM	0.701
NileTMRG	0.709
MamaEdha	0.749
ECNU	0.778
Uwaterloo	0.78
Turing	0.784
**BDPT**	**0.799**

## Data Availability

The data and the authors' source code used to support the findings of this study will be available at https://alt.qcri.org/semeval2017 (semeval2014) and https://gitee.com/hzxylwf/model.
